The article "Local anesthetic lidocaine-encapsulated polymyxin–chitosan nanoparticles delivery for wound healing: in vitro and in vivo tissue regeneration" was retracted in 2023. Reasons: lack of ethics approval or compliance; concerns about the data; concerns about the results or conclusions; concerns about the citations.

# Local anesthetic lidocaine-encapsulated polymyxin–chitosan nanoparticles delivery for wound healing: *in vitro* and *in vivo* tissue regeneration

**DOI:** 10.1080/10717544.2020.1870021

**Published:** 2021-01-27

**Authors:** Yanyan Qi, Xiangyan Yao, Xianhui Du, Songtao An

**Affiliations:** a Department of Anesthesiology, Henan Province People’s Hospital, Zhengzhou, China; b Department of Cardiology, Fuwai Central Cardiovascular Hospital, Henan Provincial People's Hospital, Zhengzhou, China

**Keywords:** Lidocaine chloride, chitosan/polymyxin B, wound healing, *in vivo* mouse model

## Abstract

In relieving local pains, lidocaine, one of ester-type local anesthetics, has been used. To develop the lidocaine membranes of enhanced local anesthetic effects, we have designed to establish the composition of wound dressings based on lidocaine chloride (LCH) (anesthetic drug)-loaded chitosan (CS)/polymyxin B sulfate (PMB). The LCH membranes (LCH-CS/PMB) was fabricated by the LCH oxide solutions within the CS/PMB matrix. The influences of different experimental limitations on CS/PMB membrane formations were examined. The double membrane particle sizes were evaluated by scanning electron microscopy (HR-SEM). Additionally, antibacterial efficacy was developed for gram-positive and negative microorganisms. Moreover, we examined *in vivo* healing of skin wounds formed in mouse models over 16 days. In contrast to the untreated wounds, rapid healing was perceived in the LCH-CS/PMB-treated wound with less damaging. These findings indicate that LCH-CS/PMB-based bandaging materials could be a potential innovative biomaterial for tissue repair and regeneration for wound healing applications in an animal model.

## 1. Introduction

An injury to the skin caused by a cut, blow, or any other impact resulting in laceration or breaking of skin is termed as a wound. Wound causes a disturbance in the defense mechanism of the skin by disrupting the epidermis (Long et al., 2018; Beyene et al., 2020; Hou et al., 2020), mucous membrane, or underlying deep tissues of the skin. According to WHO and worldwide wound incidence 2007 reporting, post-operative wounds account for the highest ratio of mortalities and infections as compared to other types of wounds. Postoperative surgical site infectious wounds may arise at the site of surgery after a month of an operation or within a year in the case of implants and infections related to the implant. Surgical site infections (SSIs) account for serious health-related complications along with economic burden, extended hospitalization, morbidity, and mortality (He et al., 2020; Liang et al., 2020; Zhang et al., 2020; Zhao et al., 2020). Surgical wound healing is a series of complex biological process that is activated by vascular constriction initiated by wounded and traumatized vessel results from myogenic spasmodic contractions of smooth muscles, localized autacoids factors from wounded tissues and involvement of nerve reflexes. After constriction of smooth muscles, the wound is often sealed with platelet plug and after stoppage of bleeding, pro-inflammatory cells migrate to the wound site and initiates inflammation. Growth factors are helpful in proliferation, restoration of skin structure, eradication of pathogenic attack, and remodeling at the site of injury (Liu et al., 2018; Deal et al., 2020; Kalantari et al., 2020).

The article "Local anesthetic lidocaine-encapsulated polymyxin–chitosan nanoparticles delivery for wound healing: in vitro and in vivo tissue regeneration" was retracted in 2023. Reasons: lack of ethics approval or compliance; concerns about the data; concerns about the results or conclusions; concerns about the citations.

Surgical site infections can be reduced with early healing but this can be hampered in the presence of risk factors like diabetes, obesity, smoking, and staphylococcus bacteria obstructing the epithelial growth, collagen production, and delayed healing. First line therapy for SSI, against *S. aureus*, include antibiotics among which cephalosporins are the drug of choice with chances of allergic reaction with this therapy (Bakshi, 2017; Nethi et al., 2019; Son et al., 2019). Bypassing the antibiotic therapy due to immense side effects, the treatment of SSIs can be successfully achieved with the local application of an ideal surgical dressing. Many chitosan and alginate-based surgical dressings, hydrogels, membranes, scaffolds, and sponges have been reported for surgical infections and are commercially available (Raja & Fathima, 2018; Memic et al., 2019; Şen et al., 2019). The use of polymyxin B (PMB) membranes formulations to heal serious burn and bone tissue injuries has been reported earlier. The CS/PMB membranes is easy to deliver, biocompatible, and biodegradable; additionally, it has low toxicity. The membranes compositions and thin films have antibacterial properties with low damage clearness capacity and high stability (Yu et al., 2016; Sekhon & Sen Gupta, 2018).

Among all commercially available dressings, the porous dressings are more popular owing to their moist nature and efficient wound healing capacity (Deal et al., 2020). An ideal wound dressing for SSI must be compatible with tissues, easily applicable on the wound, moisturized enough to induce healing, mucoadhesive to bind to the application site and antimicrobial to hamper bacterial proliferation and colonization. It may also accelerate hemostasis and tissue regeneration (Liu et al., 2018). The advent of nanotechnology has opened new avenues for designing innovative and efficient therapies to overcome the barriers faced by conventional therapies (Huang et al., 2018; Zhong et al., 2019; Alqahtani et al., 2020; Wang et al., 2020; Faraji et al., 2021). Thiolation of the polymers is a novel approach for improving the healing properties of polymers and alleviating associated side effects. Thiolated polymers are reported to have superior mucoadhesion, *in situ* gelling, poly glycoprotein (P-gp) enzyme inhibition, better control over drug release, and various other biological applications via nanotechnology chitin-covered LCH have also demonstrated promising wound management (Vellayappan et al., 2016; Han et al., 2019; Preman et al., 2020).

The article "Local anesthetic lidocaine-encapsulated polymyxin–chitosan nanoparticles delivery for wound healing: in vitro and in vivo tissue regeneration" was retracted in 2023. Reasons: lack of ethics approval or compliance; concerns about the data; concerns about the results or conclusions; concerns about the citations.

In this study, we aimed to develop wound bandages based on CS/PMB and LCH. The first step involved the fabrication of LCH inside the CS/PMB matrix (LCH-CS/PMB) by CS/PMB as an important agents. Further, the surface of LCH was modified by adding CS/PMB (LCH-CS/PMB). The CS and PMB and LCH-CS/PMB were subsequently covered with cotton fabrics to generate the final composites. The wound bandaging studies were performed with the CS, PMB and LCH-CS/PMB composites utilizing antimicrobials in vitro and in vivo animal models.

## 2. Experimental section

### 2.1. Materials

LCH oxide solutions, Polymyxin B (Mn = 80,000), Chitosan (medium molecular weight) and 3-(4,5-dimethylthiazol-2-yl)-2,5-diphenyltetrazolium bromide (MTT) were acquired from TCI, China. Luria broth and agar-agar were purchased from J&D, China. Bacterial strains of *S. aureus* and *E. coli* were obtained from our institutions. Cotton fabrics were obtained from local suppliers. All chemicals and reagents were used without further purification.

### 2.2. Fabrication of LCH-CS/PMB membranes scaffolds

Two polymer solutions were prepared based on a previously established method. In a brief, 10 wt% of PMB diluted in hexafluoroisopropanol (HFIP)/dichloromethane (DCM) (1:3) mixture and LCH was applied to the PMB solution at 2 wt% by stirring for 24 h. Afterwards, 8 wt.% chitosan solution was dissolved in the DCM/trifluoroacetic acid (TFA) combination (3:7), and 1 wt.% lid was submerged into the CS solution by mixing for 12 h.

### 2.3. Characterization of CS/PMB and LCH-CS/PMB

Scanning electron microscope (SEM) was performed to study the morphology of bandages, whereas, transmission electron microscopy (TEM) was employed for the analysis and size determination of LCH-CS/PMB. The analysis was performed using (FEI Nova Nano SEM 450, USA) equipped with TEM. Samples were carefully placed on the carbon-coated copper grid and followed by smudging with a drop of 1% ammonium molybdate solution. The particle size, zeta potential and PDI of the LCH-CS/PMB was measured using Nano-ZS (Malvern Instruments, Inc., MA).

### 2.4. Synthesis of CS/PMB and LCH-CS/PMB nanocomposites for bandaging

A nanocomposite of CS/PMB and LCH-CS/PMB for bandaging was fabricated by the DIP coating method. Briefly, cotton fabric was dished into the CS/PMB and LCH-CS/PMB solution, removed, and dehydrated at ∼60 °C for 24 h. The moisture contents of the CS/PMB and LCH-CS/PMB matrix were examined. The samples were accurately weighed and subsequently dehydrated in a hot-oven for 5 h. The dehydrated fabrics of cotton were desiccated for 24 h to remove moisture and weighed again. The moisture contents of the CS/PMB and LCH-CS/PMB were calculated using a previously reported protocol (Hoque et al., 2017; Muhamed et al., 2019; Liang et al., 2020).

The article "Local anesthetic lidocaine-encapsulated polymyxin–chitosan nanoparticles delivery for wound healing: in vitro and in vivo tissue regeneration" was retracted in 2023. Reasons: lack of ethics approval or compliance; concerns about the data; concerns about the results or conclusions; concerns about the citations.

### 2.5. Antibacterial properties of CS/PMB and LCH-CS/PMB

*In vitro*, the antibacterial efficacy of the bandage was determined by zone inhibition method. The mice were anesthetized by using chloroform, and the wound was created by sterilized needles. The sterilized swab was immediately placed on wound thus carrying wound exudates along with it and these carried wound exudates were cultured in LB broth. Following dissolution, the broth was incubated at 37 °C for 24–48 h. Bacteria were then streaked on LB agar plates separately for determination of shape and biochemical assays including gram staining, catalase, coagulase, and oxidase (Mohan et al., 2018; Sathiya Kamatchi et al., 2020; Sonamuthu et al., 2020). The cultured plates were treated with both bandages, and zones of inhibition were measured to see the antibacterial effect.

### 2.6. Animal experiments of the wound bandaging model

The animal experiments were performed according to the guidelines of the Department of Cardiology, Fuwai Central Cardiovascular Hospital, Henan Provincial People's Hospital, Zhengzhou 45000, China. Sprague-Dawley rats aged 4 weeks and weighing 200 g were used. The rats were anesthetized by injecting ketamine (30 mg/kg) and xylazine (4 mg/kg). The upper phase of the rat’s hair was detached and the specific sites were marked by skin hygienic through the soul. A 1.5-cm wide skin damage was created in the dorsum of the rats using operating scissors and tongs. The wounds were covered with the baseline damage and used as the negative control (Group I), membranes-loaded bandaging (Group II), CS/PMB (Group III), and LCH-CS/PMB (Group IV). The extent of wound closure was analyzed by drawing the wound boundary at the end of 0, 4, 8, and 16 days. The wounds closure was expressed in mm^2^. The wounds area was calculated using previously reported methods.

### 2.7. Statistical analysis

All inventory data are uttered as the mean ± standard deviations. Significant changes among groups were examined using one-way examination of modification, and changes for separate groups were dogged using Student’s *t* tests. The outcomes were observed as a significant differences when *p* < 0.05.

The article "Local anesthetic lidocaine-encapsulated polymyxin–chitosan nanoparticles delivery for wound healing: in vitro and in vivo tissue regeneration" was retracted in 2023. Reasons: lack of ethics approval or compliance; concerns about the data; concerns about the results or conclusions; concerns about the citations.

## 3. Results and discussion

### 3.1. Fabrication and characterization

By employing an easy and effective method to fabricate LCH, this study aimed at using CS/PMB as a stabilizing agents as well as a membranes system for the encapsulation of LCH. To avoid the clusters collisions and their growing into macro nanoparticle, the hydroxy fragments of CS/PMB interact with the LCH and aid in steadying them and preventing their agglomeration and further proliferation. The graphical representation of the generation and anchoring of LCH within a CS/PMB membranes matrix is depicted in Figure 1. The morphology was observed by SEM. (Figure 2(A,B)). The SEM images show spherically shaped LCH. The SEM images correspond to the DLS analysis results. The time-dependent difference in DLS analysis shows the particle size and diameters of the nanoparticles. The role of CS/PMB is to stabilize the nanoparticle formation and provide the base matrix for the membranes.

**Figure 1.** Probable schematic structure of LCH membranes (LCH-CS/PMB), lidocaine chloride (LCH)-loaded chitosan (CS)/polymyxin B sulfate (PMB). in the wound healing process.

**Figure 2.** Morphological characterization of developed CS/PMB and LCH-CS/PMB. SEM image showing the morphology of (A) CS/PMB and (B) LCH-CS/PMB.

### 3.2. Fabrication of CS/PMB and LCH-CS/PMB nanocomposites for bandaging

Cotton fabrics were used as permeable, sustainable substrates for preparing CS/PMB and LCH-CS/PMB nanocomposites. It has been preferred over other kinds of cotton because of its intrinsic properties, natural abundance, comfort, hydrophilicity, and higher heat conduction. The cotton fabrics were dished into the CS/PMB and LCH-CS/PMB solutions and dehydrated at 55 °C. The interactions amid the cotton fabrics and colloidal solutions resulted in physicochemical absorption of the gels on the surface of the cotton. The range of the cottons varied from 0.9. to 3.1% dips of coating enhanced from 1 to 4. It was witnessed that the bandaging showed a little improved flexibility with increase in the membranes content (Mohamed Subarkhan et al., 2016; Subarkhan & Ramesh, 2016; Mohamed Kasim et al., 2018).

### 3.3. LCH-CS/PMB surface morphology

The surface morphology of the bandages was examined by SEM. The SEM images in Figure 2 show the uncovered fabric form as well as the smooth surface of the fabricated LCH-CS/PMB. The additions of CS/PMB-to-CS/PMB persuades significant differences in the superficial morphology of the covered fabrics with an intricate shell-like system on the surfaces. CS/PMB enhances the rigidity and flexibility of the bandaging, though the tacky nature facilitates relaxed elimination from the wounded sites. After the releases of LCH, the morphological observations showed larger variations than those prior to release. The SEM images show the effectiveness of LCH crystals on the wounded sites. After the release of LCH, the bandage surface became rigid, rough, and flexible (Jahan et al., 2019; Silva et al., 2020; Synytsya et al., 2020).

The article "Local anesthetic lidocaine-encapsulated polymyxin–chitosan nanoparticles delivery for wound healing: in vitro and in vivo tissue regeneration" was retracted in 2023. Reasons: lack of ethics approval or compliance; concerns about the data; concerns about the results or conclusions; concerns about the citations.

### 3.4. Mechanical properties

The mechanical properties of membranes and nanocomposite are critical for successful dressing applications in order to confirm the integrity of the membranes (Nandi et al., 2019; Sun et al., 2020; Yin et al., 2020). The mechanical properties for pure materials (LCH-CS/PMB), as prepared CS/PMB and LCH-CS/PMB are shown in Figure 3(A). The addition of LCH to the LCH-CS/PMB had a variable influence on tensile strength and the overall elongation. The CS/PMB and LCH-CS/PMB exhibited a tensile strength of 2.2 ± 0.6 and 2.9 ± 0.4 MPa, respectively, which was sufficient for tissue covering the wound (Figure 3(B)). The increased compressive strength means that the samples are more fragmented. These findings have shown that the composites CS/PMB has strong surface strength suited for therapeutic use. The break elongation values represent the nGel and CS/PMB bandage versatility. Pure LCH, CS/PMB, and LCH-CS/PMB, the as-prepared CS/PMB exhibited an elongation in the range from 20 to 50% at the fracture points (Figure 3(C)). Figure 3 also shows that the tensile strength increased with an increase in Ce concentration. The result of the tensile modulus (Figure 3(D)) was consistent with the stress test. Overall, CS/PMB demonstrated higher tensile modulus and elongation than LCH, CS/PMB and LCH-CS/PMB, however it exhibited lower maximum strength. Therefore, flexibility would be an important consideration for the application of LCH-CS/PMB nanocomposites for various types of wound surface.

**Figure 3.** Mechanical properties comparison of (A) Stress–strain curve. (B) Tensile strength. (C) Elongation. (D) Tensile modulus of LCH, CS/PMB, and LCH-CS/PMB nanocomposite.

### 3.5. Biodegradation and swelling studies

Membranes s have become the subject of improvement for use in many applications (Rameshbabu et al., 2018). The percentage weight loss (Figure 4(A)) revealed limited degradation of the LCH-CS/PMB bandages. All the as-fabricated bandages showed a degradation of 24 to 27% (1 day), 39 to 48% (4 days) and 75 to 84% (7 days) after immersion in PBS medium, respectively. The presence of LCH reduced the degradation rate in the composite bands. The interaction of LCH, CS/PMB and LCH-CS/PMB bandages can be due to this. However, the as-manufactured bandage has been in vitro deteriorated although its features and shape have remained unaltered even after the 7th day. After 1, 4, and 7 days of incubation in PBS medium, swellings of the CS/PMB and LCH-CS/PMB dressings were examined (Figure 4(B)). Figure 4(B) suggested that LCH-CS/PMB exhibited higher swelling capacity compared to pure CS/PMB membranes bandages. Furthermore, even after LCH were introduced, the nGel and LCH-CS/PMB bands displayed similar swelling behavior. The existence of LCH nanoparticles of different dimensions, morphology and surface charges will lead to an improvement in the swelling capacity of LCH-CS/PMB. Furthermore, nanoparticles forming LCH may cause the LCH-CS/PMB to expand, widening pores, and the open spaces in LCH-CS/PMB, thus absorbing more water.

The article "Local anesthetic lidocaine-encapsulated polymyxin–chitosan nanoparticles delivery for wound healing: in vitro and in vivo tissue regeneration" was retracted in 2023. Reasons: lack of ethics approval or compliance; concerns about the data; concerns about the results or conclusions; concerns about the citations.

**Figure 4.** (A) Biodegradation and (B) Swelling ratio as-fabricated bandages of CS/PMB and LCH-CS/PMB nanocomposite using different days (1, 4, and 7) of activity.

### 3.6. Antibacterial and cell viability analyses

The antibacterial properties of the fabricated CS/PMB and LCH-CS/PMB dressings were investigated using *S. aureus* (gram-positive microbe) and *E. coli* (gram-negative microbe), and the results are shown in Figure 5(A,B). In our previous studies, the LCH-CS/PMB dressings exhibited higher antibacterial activity with both microbes compared to LCH-CS/PMB. The bacterial property of LCH-CS/PMB was reduced by the presence of free LCH-CS/PMB.

**Figure 5.** Antibacterial and cell viability examinations. (A, B) Colony formation of *S. aureus* and *E. coli*. (C, D) Cell viability of CS/PMB and LCH-CS/PMB. The experiments were repeated three times. Values are expressed as the mean ± SD. *p < 0.05, **p < 0.01.

The outcomes of cell viability established that LCH (positive control) and CS/PMB (control) did not demonstrate any harm on days 1, 3, and 7 in development with NIH-3T3 fibroblasts (Figure 5(C,D)). The synthesized LCH-CS/PMB dressings showed ∼75% viability after day 1 of culture, which further increased up to ∼93% after 3 and 7 days of development. The reduced cell viability on day 1 was due to the presence of free CS/PMB with the NIH3T3 fibroblasts. After day 1, the remaining viable fibroblasts multiplied, consequently improving the viability.

### 3.7. In vivo examination of LCH

The results of the in vivo investigation of the CS/PMB and LCH-CS/PMB are shown in Figure 6. The CS/PMB and LCH-CS/PMB dressings displayed outstanding wound healing properties after 0, 4, 8, and 16 days, compared to saline treatment (Figure 6(A)). The reduction in wound damage in mouse models at different periods (0, 4, 8, and 16 days) can be seen in the Figure 6. The treatment with fabric control displayed ∼50% wound reduction after day 16, while coating with membranes bandaging resulted in 70% reduction. The LCH-CS/PMB-treated wound attained 80% closure on day 16. LCH-CS/PMB treated mice had almost complete wound closure after day 16. This improved rate of wound closure was attributed to the rapid healing properties of the LCH released from the bandaging in the presence of CS and PMB (Figure 6(B)). The LCH released from the membranes s slowly changed the physiological conditions and interacted with specific wound sites. Further, Ce has been gambled to decrease the period for fibroblast to enter wounds. It also has excellent anti-inflammatory properties, which may enhance the re-epithelialization rate (Horii et al., 2016; Gao et al., 2017; He et al., 2019).

The article "Local anesthetic lidocaine-encapsulated polymyxin–chitosan nanoparticles delivery for wound healing: in vitro and in vivo tissue regeneration" was retracted in 2023. Reasons: lack of ethics approval or compliance; concerns about the data; concerns about the results or conclusions; concerns about the citations.

**Figure 6.** Photographs of an in vivo wound healing study. (A) Extent of closure of wounds treated with control, CS/PMB and LCH-CS/PMB. (B) Evaluation of the wound area shutter. The values are expressed as the mean ± SD. *p < 0.05, **p < 0.01.

### 3.8. Histological evaluation

Histological study is a powerful tool for observing improvement in cure and tissue regeneration. The histological based on a specified on the healing potential of damaged mouse tissue caused by the effect on the CS/PMB and LCH-CS/PMB (Figure 7) by hematoxyl and eosin (H&E). After 0, 4, 8, and 16 days, the LCH-CS/PMB displayed excellent healing as compared to the naked wound. Figure 7 shows that compact keratinocytes in the epidermis are indicated for CS/PMB and LCH-CS/PMB wounds relative to the bare wound in histological parts. Furthermore, LCH-CS/PMB also increased the healing rate of CS/PMB-coated wounds as shown in the histological micrograms. LCH nanoparticles have biocompatible and anticoagulant properties, making it an excellent candidate for wound cure, as shown in the study in vitro and in vivo. In comparison, a segment light microscopy quantitated absolute new subcutaneous tissue growth. The degree of wound closure was macroscopically calculated (Figure 7). Therefore, in vivo study of Sprague-Dawley rats confirmed the increased wound healing ability of the as-fabricated LCH-CS/PMB. The results (Figure 7) suggested that the LCH-CS/PMB nanocomposite treatment promotes significant healing through the migration of fibroblasts and appropriate development of epithelial cells, and the restoration of blood flow via training of new blood vessels. In our effort to introduce a tissue treating method, we have developed LCH-CS/PMB bandage material based on CS/PMB conjugated with LCH, which was first tested for tissue regeneration care management, to the best of knowledge.

The article "Local anesthetic lidocaine-encapsulated polymyxin–chitosan nanoparticles delivery for wound healing: in vitro and in vivo tissue regeneration" was retracted in 2023. Reasons: lack of ethics approval or compliance; concerns about the data; concerns about the results or conclusions; concerns about the citations.

**Figure 7.** Photomicrographs H&E-stained control, as-fabricated bandages of control, CS/PMB, and LCH-CS/PMB nanocomposite treated wounds.

## 4. Conclusion

Our study aimed at developing novel wound bandages by covering double membranes loaded with LCH on the surface of cotton fabrics. Herein, cotton acts as a supporting layer for the membranes. Well-dispersed LCH are generated with the stabilizing effect of CS/PMB as the membranes medium. The membranes thus formed had a size in the series of ∼10–50 nm. Together CS/PMB and LCH-CS/PMB nanocomposite bandages showed significant antibacterials properties even at low absorptions. A slow rate of releases were detected for the membranes s bandages with ∼2 µg/cm^2^ of Ce leaking out in 48 h. These low attentions of Ce are very nontoxic for the human body. The LCH-CS/PMB bandaging displayed 100% closure of full width wound by day 16, which may be because the occurrence of CS/PMB quickens in the medium, therefore assisting wounds closure. The wound bandages might be effortlessly exposed off from the wounds sites without affecting the tissues. The results of these investigations suggest that LCH-CS/PMB could be a promising wounds care management composition having effective damage and scar prevention.
